The article "The Reform of University Education Teaching Based on Cloud Computing and Big Data Background" was retracted in 2023. Reasons: unreliable results or conclusions; concerns about the data; concerns about the peer review; concerns about the citations.

# The Reform of University Education Teaching Based on Cloud Computing and Big Data Background

**DOI:** 10.1155/2022/8169938

**Published:** 2022-08-12

**Authors:** Jing Li, Lei Liu

**Affiliations:** ^1^School of Management, Hubei University of Chinese Medicine, Wuhan, Hubei 430065, China; ^2^Hubei University of Technology Engineering and Technology College, Wuhan, Hubei 430065, China

## Abstract

In the era of big data and cloud computing, traditional college teaching model needs to be revolutionized in order to adapt to the needs of the present generation. The traditional college teaching model is currently facing unprecedented severe challenges which could be optimistically considered as a huge scope of development opportunity. In order to promote the gradual transformation of college teaching toward digitization, intelligence, and modernization, this paper comprehensively analyzes the impact of science and technology on college teaching. It further encourages the omnidirectional and multifaceted amalgamation of education with big data and cloud computing technology with an objective to improve the overall teaching level of colleges and universities. In order to realize the accurate evaluation of university teaching reform and improve teaching quality, the study presents an evaluation method of university teaching reform based on in-depth research network. Then, it further analyzes the main contents of university teaching reform, establishes the evaluation department of university teaching reform, and then establishes the evaluation model of university education reform. This is achieved by analyzing the relationship between university education reform and indicators using in-depth learning network followed by the development of simulation experiments pertinent to evaluation of university education reform. The results show that this method is helpful in improving the teaching quality.

## 1. Introduction

The rapid development of modern information and communication technology, such as 4G, 5G, computer, big data, and cloud computing, continues to accelerate the arrival of the era of big data and cloud computing [1]. At the same time, the era of big data and cloud computing is also the driving force of large-scale changes in the field of information technology, which has an increasing impact on modern people's daily life and labor training [2]. In recent years, with the accumulation of big data and the calculation of cloud cover, the national level has been listed as a key project of national construction, and a series of corresponding supporting policies and measures have been issued [3]. The development of big data and cloud computing industry does not rely on high-quality technical talents. As the main battlefield for the cultivation of reserve talents for socialist modernization, universities shoulder the great responsibility of cultivating the best talents for the society and the country [4].

Big data processing and cloud technology provide a reliable guarantee for improving the quality of talent training. In the context of big data processing technology and cloud volume, the level of public access to information resources and the frequency and depth of contact between universities, public enterprises, and a series of users have been greatly improved, and higher education institutions have more fully considered the basic training requirements of employers [5]. This makes it possible to adjust the training plans and programs in time, make major changes to the educational contents, train high-quality talents for enterprises more specifically, and improve their quality and efficiency through cooperation between training institutions and integration into production activities [6]. At the same time, big data processing technology and “cloud” provide a good foundation for the development of educational modernization and internationalization, rapidly expand new teaching forms such as Q & A and micro courses, constantly change traditional educational ideas, and promote the open allocation of educational resources [7].

Big data processing technology and cloud technology pose a severe challenge to the teaching reform of colleges and universities. Under the traditional school teaching mode, teachers have long been the main speaker in the curriculum, students are relatively passive, and teachers occupy a prominent position [8]. At the same time, under the influence of big data technology and cloud computing technology, the role of teachers has changed from lecturer and course leader to instructor and organizer of teaching activities aimed at cultivating students' skills and knowledge, that is, students of different disciplines [9].

Therefore, in the era of big data processing technology and cloud computing technology, the traditional and overall teaching concept can no longer meet the basic requirements of modern teaching work. The teachers' teaching concept and knowledge coverage and structure need to be updated [10]. It is absolutely necessary to create a favorable environment for student-centered subject teaching, explore students' advantages, and establish a teaching system focusing on low education level [11]. Therefore, big data processing and cloud technology have brought challenges to university teaching. College teaching reform strategy is based on big data technology and cloud computing technology. The advent of the era of big data and cloud computing has brought broad opportunities and severe challenges to the modernization and development of teaching work in colleges and universities in China. To effectively improve the teaching quality and efficiency of colleges and universities and promote the development of government and social talents, a new education system based on big data technology and cloud computing technology must be established to promote the ultimate goal of reform [12].

Various studies have been conducted in education sector involving deep learning techniques. For example, the study in [13] highlighted the role of deep learning in automating the process of intellectual education on the basis of image detection techniques. The study proposed a customized intelligent education framework incorporating deep learning techniques. The system provided relevant resources of the evolution of the ecosystem to learners as per their choices and perceptions. The study in [14, 15] used a gamification tool that helped to promote commitment and encourage motivation of students. The gamified application contributed immensely to the pro-deep-learning approaches which exposed the students' private learning actions to their friends making the entire experience worthwhile. The students' satisfaction level and their promotion of deep learning strategies related to behavioral aspect were achieved. Hence, it is obvious that deep learning techniques have immense popularity in academic implementations.

## 2. Related Work

In the era of big data and cloud cover, data collection is a real-time, consistent, and natural method, which can collect the data of learning process in real time and continuously, such as browsing tracking, browsing time, reply time, correctness of answers, teacher-student interaction, and student interaction [16]. The data structure of education data is more complex, including structured data, such as student performance, student facsimile information, student attendance records, book borrowing records, and student employment rate; there are also unstructured data, such as videos, pictures, lesson plans, teaching software, and documents, which makes the analysis and processing of data more complex, and the comprehensive and huge data lead to more in-depth application of education data [17].

Universities should fully understand the value and content of new teaching modes such as “micro course” and “monthly course,” make full use of petroleum computing platform and computer Internet technology, summarize their existing teaching resources, and take them as the basis of education and teaching reform [18]. In particular, the diversified teaching mode should be combined with multiple modes such as hierarchical group training, specific task teaching, class reform, and artificial intelligence teaching and closely combined with the five cycles of teaching, training, management, assessment, and assessment [19]. In the process of applying the above diversified learning mode, we should actively change students' traditional learning habits, so that they can use scientific computers and intelligent mobile communication terminals in the learning process, and give full play to the advantages of large database and cloud computing platform [20]. Then, teachers analyze the results through a wide range of information platforms, find out the problems faced by students, and formulate strategies to solve them in time.

As one of the core contents of talent training in colleges and universities, teachers' comprehensive quality and professional quality directly affect the quality of talent training [21]. Therefore, teachers are an important and indisputable link in the process of higher education teaching reform. In the era of big data, with the rapid renewal of knowledge and easy access to property, the authority of traditional teachers is weakening, which requires them to constantly improve their knowledge system and skills and improve their comprehensive quality [22]. At the same time, schools need to improve the importance of teacher training by closely connecting teachers' work with a wider data-based education management platform, so as to effectively integrate education teaching, management, and scientific research. A large database is used to record the growth and training of university teachers before and after training and provide scientific suggestions for their development, thereby finally continuously improving the overall level of college teachers and promoting the early completion of the task of educational reform [23, 24].

The study in [25] used deep learning techniques to predict students' performance in higher education. This helped students in selecting courses of study and also develop better future education plans. The proposed method used deep neural network for prediction based on informative data as a feature having respective weights. The results of the model were evaluated on the basis of mean absolute error (MAE) and root mean square error (RMSE) and accuracy. The study in [26, 27] used deep learning technique to analyze students' interest in physical education (PE) using convolutional neural network technique (CNN). The case of solid ball throwing was considered, and the students' interest, learning ability, and physical quality were investigated using a questionnaire based approach. The use of deep learning resulted in significant improvement in the teaching of physical education.

College teaching evaluation is an important content to evaluate the teaching level of students and teachers. It generally includes the evaluation of teachers' teaching effect and the evaluation of students' teaching effect. However, the traditional teaching evaluation generally adopts the unified evaluation method, and the attention of process evaluation and comprehensive evaluation is low [28]. The results are not accurate for both teachers and students. In view of this, in the process of promoting the reform of the education system, we should actively use big data and cloud technology to build a multidimensional education evaluation system. In terms of teacher evaluation, it integrates teacher evaluation, school management evaluation, self-evaluation, student evaluation, etc. In this process, each assessment participant must upload relevant data to a wider database and then comprehensively evaluate the learning level through cloud assessment and big data analysis methods. In the student assessment, we must accurately record the learning time, learning content, learning methods, learning track, learning ability, examination results, classroom results, etc.

## 3. Exploration of Educational Reform Taking Online Teaching as an Example

Due to the impact of Newcastle pneumonia, all universities have postponed the start of spring study and launched on-the-job training programs. The main task of network teaching in colleges and universities is to improve the quality of network teaching. Therefore, it is of great significance to study effective evaluation methods of university education reform. Studying the evaluation methods of teaching reform in colleges and universities can strengthen the management of network teaching quality and improve the quality of network teaching.

Deep learning network is an extension of neural network, which has strong feature learning ability, and the learned features can restore the characteristics of data, and has good visualization and data classification effect. DBN is an unsupervised learning algorithm, which is used to initialize DBN layer by layer. The time complexity and network size of optimized DBN weights are linearly related to the depth. We take the simple single layer problem as the starting point to solve the problem of complex depth layers constructed by single layer and reduce the training difficulty of deep learning network.

DBN model is a deep learning model that has gained immense momentum due to its ability to implement a successful and efficient learning technique that stacks simpler models such as Boltzmann machines (BMs). The DBN based deep neural network model improves the performance of the model by eliminating possibilities of overfitting, thereby improving model generalization. This network provides the ability to perform feature selection and extraction without the need for explicit ad hoc elaborations. It also generates samples based on features that the model learns during the training phase, being a generative model. The study in [29, 30] used a DBN model to understand schizophrenia pathology wherein a DBN based deep learning model was used to extract features from brain morphometry data. This helps to investigate its performance discriminating healthy controls from patients suffering from schizophrenia.

The factors influencing the educational teaching reform are teaching preparation, content, methods, resources, and effects. The evaluation system of higher education teaching reform is shown in Table 1. The secondary indicators are numbered *x*_*i*_, *i* = 1,2,…, 20.

Teaching preparation is the key to the reform of university education, and the preparation of online teaching is more complicated than offline teaching; there are many uncertainties in the implementation of online teaching, including the stability of the teaching platform and students' self-management level. The content of teaching is a prerequisite for students to achieve the desired learning effect, and it is necessary to highlight the key points and difficulties of teaching content to enable students to fully understand the knowledge of professional courses and improve their learning efficiency.

Deep belief network (DBN) model is a series of top-down finite Boltzmann models (FBM). The preliminary preparation of multilayer RBM based on runaway greed shows that each layer of RBM must be trained with weights in order to bind the hidden layer to the high-level data specified in the visible layer. The non-prefabricated DBN model is a reasonable choice of the initial value of the DBN model of the network, and then the traditional callback method is used to optimize the network parameters, which does not produce the relevant problems of local optimal solution [31–33]. The module based on cross bar array is shown in Figure 1 [17]. A four-layer computing model including response and emotion engine is proposed. From the perspective of semantic representation, these symbolic models are sufficient [18]. Such models are reviewed. However, [19] believes that these models are overdesigned and too complex, so they are not suitable for intelligent control.

In order to be able to implement intelligent emotion networks of artificial emotions in concrete intelligent systems, it is necessary to reduce the complexity of emotion models, and this new approach to emotion modeling emerged. In [20], a relatively simple emotion model as shown in Figure 2 was designed based on a specific task and environment, using a bottom-up analysis approach to move from the abstract to the concrete and to capture the main factors that affect the system performance. The model considers sensation, perception, emotion, and hormone systems, and emotion exhibits the following four characteristics:

1. Emotion is measured numerically; i.e., it can be expressed as a positive or negative number.
2. A certain emotional state lasts for a certain period of time, and sudden changes between different emotions are not allowed, especially for two very different emotions.
3. The generation of a certain emotion is not only dependent on the current feeling but also related to its recent emotional state.
4. The current emotional state can influence or even distort the subject's perception.

The model contains four basic emotions, namely, happiness, sadness, anger, and fear, all closely related to the state of the subject and the environment in which he or she lives. An et al. [21] pointed out that there are two problems with pre-emotional modeling (e.g., OCC):

1. Emotions evaluate something as an absolute good/bad concept that changes too quickly.
2. When emotions evaluate the degree to which something satisfies multiple goals, they usually consider the degree to which each goal is satisfied separately and lack integration.

Therefore, they proposed a fuzzy model of emotion based on fuzzy goal satisfaction, influence level, and fuzzy mapping of events to goals. The structure is the same as Gadanho's model, but fuzzy reasoning is used for the two aspects of external stimuli leading to emotion generation and emotional states leading to behavior, solving the two previously mentioned problems. Reference [22] also used fuzzy logic to build a model based on perception (feeling), emotion (mood), and affect, arguing that a mathematical model can be used to represent the interactions between the three. Reference [23] proposed a computational model of emotion from the perspective of intelligent speech signal processing, whose basic structure follows the mainstream theory of psychology from sensory stimulus to emotion to behavior.

Although the above models are very imperfect with respect to the rich emotional life of humans, their simple structure allows them to be applied in various intelligent systems.

In order to ensure that the deep-rooted belief network model conforms to the characteristics of the university education reform evaluation system, at the first level, Gauss–Bernoulli RBM is used to map the characteristics of the university education reform evaluation system into a binary state, and all other RBM levels abstractly describe the basic relationship between Bernoulli–Bernoulli characteristics. We use the softmax classifier to execute the MOS (mean opinion score) function. Joint probability distribution formula of Neos and other hidden layers in depth network model are as follows:

(1) $$\begin{array}{c} p\left(v,h^{1},h^{2},\ldots ,h^{s}\right)\;=p\left(v|h^{1}\right)p\left(h^{1}|h^{2}\right)\cdots p\left(h^{s-2}|h^{s-1}\right)p\left(h^{s-1}|h^{s}\right), \end{array}$$

where *s* is the number of hidden layers.

When *s* = 2, this means that the two learning processes of Bernoulli–Bernoulli RBM stratification and greed are also trained into two or more deep belief screening network models. Assuming that the number of nodes *v* and the number of nodes in the layer *h*^2^ are the same, the joint probability of visible layer and hidden layer can be obtained in the form of sampling process equation:

(2) $$\begin{array}{c} p\left(h|v^{0}\right)⟶h^{0}\Rightarrow p\left(v|h^{0}\right)⟶v^{1}\\ \cdots p\left(h|v^{n}\right)⟶h^{n}\Rightarrow p\left(v|h^{n}\right)⟶v^{n+1}\cdots , \end{array}$$

(3) $$\begin{array}{c} p\left(v,h^{1},h^{2};\theta \right)=p\left(h|v^{1};W^{1}\right)p\left(h^{1},h^{2};W^{2}\right), \end{array}$$

(4) $$\begin{array}{c} \left\{\begin{array}{c} p\left(v_{i}=1|h^{1};W^{1}\right)=f\left[\sum_{j}W_{ij}^{1}h_{j}^{1}\right],\\ p\left(h^{1},h^{2};W^{2}\right)=\frac{1}{Z\left(W^{2}\right)}\exp\left(h^{1T}W^{2}h^{2}\right). \end{array}\right. \end{array}$$

The initial state of the visual layer is *v*^0^; the state of the visual layer reconstructed by the nth sampling is *v*^*n*^, *v*^*n*^; i.e., the state of the visual layer reconstructed by *h*^*n*−1^ is *v*^*n*^; the state of the hidden layer composed of samples is *h*^*n*^; the random variable is *Z*; the Sigmoid function is *f*; the number of iterations is *T*; the bias of each layer is set to 0; and the parameters of the DBN model can be simplified to *θ*={*W*^1^, *W*^2^} at this time. The weights *W*^2^ between the hidden layers are initialized to *W*^1^. Based on (5), the joint probability distribution *p*(*v*, *h*^1^; *θ*) shows that the in-depth learning network model conforms to the RBM joint probability distribution *p*(*v*, *h*^1^; *W*^1^), as follows:

(5) $$\begin{array}{c} p\left(v,h^{1};\theta \right)=\sum_{h^{2}}p\left(v,h^{1},h^{2};\theta \right)n\times \sum_{h^{2}}p\left(h^{1},h^{2};W^{2}\right)n=\prod_{i}\frac{\text{exp}\left[v_{i}\sum_{j}W_{ij}^{1}h_{j}^{1}\right]}{1+\text{exp}\left[\sum_{j}W_{ij}^{1}h_{j}^{1}\right]}\times \frac{1}{Z\left(W^{2}\right)}\prod_{i}\left\{1+\exp\left[\sum_{j}W_{ij}^{2}h_{j}^{1}\right]\right.. \end{array}$$

Equation (5) can be simplified to the following equation according to *W*_*ij*_^1^ = *W*_*ji*_^2^, *Z*(*W*^1^) = *Z*(*W*^2^):

(6) $$\begin{array}{c} p\left(v,h^{1};\theta \right)=\frac{1}{Z\left(W^{1}\right)}\prod_{i}\exp\left[v_{i}\sum_{j}W_{ij}^{1}h_{j}^{1}\right]\\ =\frac{1}{Z\left(W^{1}\right)}\exp\left[\sum_{ij}W_{ij}^{1}v_{i}h_{j}^{1}\right]\\ =p\left(v,h^{1};W^{1}\right). \end{array}$$

According to (6), the DBN model *p*(*h*^1^, *W*^1^) is consistent with the RBM's *p*(*v*, *h*^1^; *W*^1^) as well; therefore, the greedy layer-by-layer pretraining steps for the existence of *s*-layer hidden depth belief network model are as follows:

  Step 1: Train the RBM to obtain the weight parameters of the bottom layer RBM *W*^1^.
  Step 2: Start training the second layer RBM, initialize the second layer weight parameters *W*^2^=*W*^1*T*^, ensure that the DBN model with two hidden layers is better than the RBM without initialization, and then train the second layer RBM by fixing *W*^1^ to make *W*^2^ optimal.
  Step 3: Continue to train the third layer RBM, initialize the third layer RBM weight parameter *W*^3^=*W*^2*T*^, train the third layer RBM to optimize *W*^3^ by fixing *W*^2^, similarly finish the last layer RBM weights for optimization, and complete the unsupervised pretraining of the whole DBN model.

At the top level of DBN model, the output layer is introduced to expand the number of classes based on softmax logistic regression and realize the evaluation of all indicators of university education reform and higher education reform. Since the score of university education reform shows that it is a multifaceted classification problem, the integration of logistic has been expanded in the process of returning to softmax [34, 35].

The state code of each neuron in the hidden layer {(*x*^1^, *y*^1^),…, (*x*^*n*^, *y*^*n*^)} and the corresponding class of each neuron are established. For the class, the mark corresponding to the characteristic class is *y*^*i*^∈ {1,2,..., *M*}, one-dimensional probability distribution matrix is as follows:

(7) $$\begin{array}{c} l_{\sigma }\left(x^{i}\right)=\left[\begin{array}{c} p\left(y^{i}=1|x^{i};\sigma \right)\\ p\left(y^{i}=2|x^{i};\sigma \right)\\ ...\\ p\left(y^{i}=M|x^{i};\sigma \right) \end{array}\right]=\frac{1}{\sum_{j=1}^{M}e^{\sigma_{J}^{T}x^{i}}}\left[\begin{array}{c} e^{\sigma_{1}^{T}x^{i}}\\ e^{\sigma_{2}^{T}x^{i}}\\ ...\\ e^{\sigma_{M}^{T}x^{i}} \end{array}\right],\\ \sigma =\left[\begin{array}{c} \sigma_{1}^{T}\\ ...\\ \sigma_{M}^{T} \end{array}\right]. \end{array}$$

Types and models of matrix parameters is *M* × *N*; and then enter the feature size. The softmax cost regression function shows

(8) $$\begin{array}{c} J\left(\sigma \right)=-\frac{1}{N}\left[\sum_{i=1}^{n}\sum_{j=1}^{M}1\left\{y^{i}=j\right\}\log\frac{e^{\sigma_{J}^{T}x^{i}}}{\sum_{d=1}^{M}e^{\sigma_{d}^{T}x^{i}}}\right]=\frac{\tau }{2}\sum_{i=1}^{M}\sum_{j=0}^{N}\sigma_{ij}^{2}. \end{array}$$

By minimizing the cost function through the gradient descent, the gradient function is obtained as follows:

(9) $$\begin{array}{c} \nabla_{\sigma_{j}}J\left(\sigma \right)=-\frac{1}{n}\sum_{i=1}^{n}\left[x^{i}\left(1\left\{y^{i}=j\right\}\right)-p\left(y^{i}=j|x^{i};\sigma \right)\right]+\tau \sigma_{j}. \end{array}$$

In the case of optimizing teaching parameters, indicators will be considered according to the calculation of relevant indicators of education reform in each university, and after studying the DBN model with teaching model parameters, the most likely quality indicators will be selected as the inference results.

## 4. Experiments and Results

The online learning data provided by the university from March to August 2021 was selected as a dataset containing 5000 data samples. The online teaching quality evaluation method based on in-depth learning network and the selected indicators shown in Table 1 are used to evaluate the online teaching quality of the school. The evaluation index is divided into 10 off-campus experts who are familiar with online teaching and 5 senior teachers, with an average of the final evaluation index of each evaluation level [0-1]. Tables 2 and 3 show the reliability survey results of students' comprehensive knowledge assessment data based on cloud platform.

### 4.1. Learning and Training Performance

In order to verify the learning and training performance of the DBN model used in this application, 3000 data samples from 5000 data samples are selected as the simulation training module, the other 2000 data samples are used as the model test suite, and the data collected in the preparation process is used as the original module of model input. It can be seen from the data in Figure 1 that with the increase of the number of iterations of the DBN model construction error used in this paper, the number of iterations decreases significantly. When the number of iterations reaches 20, the DBN model simulation error stabilizes and decreases to less than 0.01. The experimental results in Figures 3 and 4 show that the model has good learning ability and small approximation error.

In order to compare the simulation results with the expected results, as shown in Table 4, they are divided into 10 groups for centralized screening from 2000 test samples. As shown in Table 4, the relative error between the conclusion drawn by the model and the expected conclusion is less than 3%, and the estimation level of the method is the same as the actual level. The experimental results show that the model has high evaluation accuracy and can be effectively applied to the evaluation of university education reform.

### 4.2. Evaluation Performance

Karl Pearson correlation coefficient and root mean square error (RMSE) are used to evaluate the convergence and instability of effective online teaching quality evaluation results. According to the actual evaluation of teaching quality, the effectiveness of this method is verified. The root mean square errors of correlation coefficient *R* and RMSE are calculated in the process of method estimation, as shown in Table 5. The analysis of the data in Table 5 shows that the correlation coefficient of this method is greater than 0.85 and RMSE is less than 0.45. The results show that the evaluation results of this method are similar to the actual evaluation level and the error is small. It can be effectively applied to the evaluation of teaching reform in colleges and universities.

From the above experiments, it can be seen that this method has a good effect in the evaluation of university education system reform. Therefore, this method is used for the evaluation of university teaching quality, as shown in Table 6. The analysis of the data in Table 6 shows that this method can evaluate the quality of university online education according to the quality index of university online education. According to this method, the quality of university network teaching is evaluated on average. According to this method, schools can evaluate lower indicators and take targeted measures to improve teaching quality.

## 5. Conclusion

With the development of cloud computing technology and big data and the update of network education technology, higher education needs to be reformed in order to obtain a new education model. In order to improve the teaching quality, this paper studies the evaluation method of college teaching reform based on deep learning network. The present study uses a DBN based deep learning model to study the evaluation method of college teaching reform. The results of the model are evaluated against the Karl Pearson coefficient and RMSE metrics which justify the superiority of the model. This method can effectively evaluate the teaching quality of top colleges and universities. In addition, teachers can also obtain classroom quality feedback, and better understand students' knowledge, so that they can comprehensively analyze and improve knowledge and improve the effectiveness of knowledge. The experimental results show that the method proposed in this paper can effectively improve the quality of education and promote the teaching reform in colleges and universities.

## Figures and Tables

**Figure 1:** Cross-array module.

**Figure 2:** Emotional model.

**Figure 3:** Learning performance of DBN model.

**Figure 4:** Training performance of DBN model.

**Table 1:** Evaluation system of educational teaching reform.

Evaluation object	Primary index	Secondary index

Teaching quality	Teaching preparation	Debug the teaching platform before implementing online teaching; set up preparation for online teaching emergencies; select the online teaching platform; remind students to prepare for class; clarify the course objectives and the actual teaching content in line
	Teaching content	Online teaching content is well organized, informative, and of high quality; the teaching content is clearly explained; highlight the key points and difficulties of the teaching content; give off-class assignments; facilitate students' understanding of the course content
	Teaching resources	Select online course video materials; select online teaching course PF; select online teaching test bank; basically achieve the purpose of online teaching, satisfaction of solving problems for students; focus on the interaction rate with students during online teaching
	Teaching effect	Stimulate students' interest in learning, class acceptance rate, students' performance in the online test; focus on students' efficiency in completing assignments in class; focus on students' opinions about online teaching

**Table 2:** Evaluation criteria of educational teaching reform.

Evaluation score	Estimated grade

>0.75	Excellent
0.5∼0.75	Good
0.25∼0.49	Fair
<0.25	Poor

**Table 3:** Investigation of the credibility of the data of comprehensive student literacy evaluation based on the cloud platform (*N* = 550).

Question	Options	Frequency	Percentage

(4) Credibility of student evaluation data based on cloud platform (single choice)	High	289	55
	Medium	188	32
	Low	55	10
	Not indicative	17	3

**Table 4:** Model test results.

Dataset	Expected output	Actual rating	Test output	Evaluation level	Relative error (%)

1	0.75	Excellent	0.81	Excellent	1.27
2	0.58	Good	0.61	Good	1.71
3	0.40	General	0.45	General	2.3
4	0.53	Good	0.56	Good	1.93
5	0.11	Poor	0.12	Poor	0
6	0.22	Poor	0.25	Poor	0
7	0.89	Excellent	0.88	Excellent	1.15
8	0.47	General	0.46	General	2.16
9	0.83	Excellent	0.82	Excellent	1.23
10	0.67	Good	0.67	Good	1.55

**Table 5:** Statistical results of *R* and RMSE.

Dataset	*R*	RMSE

1	0.93	0.26
2	0.89	0.33
3	0.88	0.45
4	0.91	0.32
5	0.92	0.31
6	0.95	0.22
7	0.89	0.34
8	0.91	0.25
9	0.92	0.33
10	0.94	0.21

**Table 6:** Online education quality assessment results.

	Level 1 indicators	Weighting of primary indicators	Secondary indicators	Secondary indicator weights	Weighting results

Teaching preparation	0.1	*X*_1_	0.3	0.65	
		*X*_2_	0.4	0.75	
		*X*_3_	0.3	0.88	
		*X*_4_	0.2	0.69	
		*X*_5_	0.1	0.55	

Teaching content	0.2	*X*_6_	0.2	0.32	
		*X*_7_	0.3	0.55	
		*X*_8_	0.4	0.68	

Teaching method	0.3	*X*_9_	0.2	0.57	
		*X*_10_	0.1	0.52	0.70
		*X*_11_	0.3	0.53	

Teaching resources	0.2	*X*_12_	0.1	0.31	
		*X*_13_	0.2	0.49	
		*X*_14_	0.1	0.88	
		*X*_15_	0.1	0.77	
		*X*_16_	0.2	0.54	

Teaching effect	0.2	*X*_17_	0.3	0.59	
		*X*_18_	0.2	0.69	
		*X*_19_	0.1	0.78	
		*X*_20_	0.1	0.89	

## Data Availability

The dataset used in this paper is available from the corresponding author upon request.
